The article "Probiotics and Functional Gastrointestinal Disorders in Pediatric Age: A Narrative Review" was published in 2022. Journal: Front Pediatr.

# Probiotics and Functional Gastrointestinal Disorders in Pediatric Age: A Narrative Review

**DOI:** 10.3389/fped.2022.805466

**Published:** 2022-02-16

**Authors:** Manuela Capozza, Nicola Laforgia, Valentina Rizzo, Silvia Salvatore, Stefano Guandalini, Mariella Baldassarre

**Affiliations:** ^1^Section of Neonatology and Neonatal Intensive Care Unit, Department of Biomedical Science and Human Oncology (DIMO), University of Bari “Aldo Moro”, Bari, Italy; ^2^Section of Neonatology and Neonatal Intensive Care Unit, Interdisciplinary Department of Medicine (DIM), University of Bari “Aldo Moro”, Bari, Italy; ^3^Department of Pediatrics, University of Insubria, Ospedale “F. Del Ponte”, Varese, Italy; ^4^Section of Gastroenterology, Department of Pediatrics, Hepatology and Nutrition University of Chicago, Chicago, IL, United States

**Keywords:** probiotics, pediatric age, functional abdominal pain, functional gastrointestinal disorders, infantile colic, irritable bowel syndrome, constipation, gastroesophageal reflux

## Abstract

Assessment and management of pain are essential components of pediatric care. Pain in pediatric age is characterized by relevant health and socio-economic consequences due to parental concern, medicalization, and long-term physical and psychological impact in children. Pathophysiological mechanisms of nociception include several pathways in which also individual perception and gut-brain axis seem to be involved. In this narrative review, we analyze the rational and the current clinical findings of probiotic use in the management of functional gastrointestinal disorders (FGID) in pediatric age, with special focus on infantile colic, irritable bowel syndrome, constipation, and gastroesophageal reflux. Some specific probiotics showed a significant reduction in crying and fussing compared to placebo in breastfed infants with colic, although their exact mechanism of action in this disorder remains poorly understood. In irritable bowel syndrome, a limited number of studies showed that specific strains of probiotics can improve abdominal pain/discomfort and bloating/gassiness, although data are still scarce. As for constipation, whilst some strains appear to reduce the number of hard stools in constipated children, the evidence is not adequate to support the use of probiotics in the management of functional constipation. Similarly, although some probiotic strains could promote gastric emptying with a potential improvement of functional symptoms related to gastroesophageal reflux, current evidence is insufficient to provide any specific recommendation for the prevention or treatment of gastroesophageal reflux. In conclusion, probiotics have been proposed as part of management of pain in functional gastrointestinal disorders in pediatric age, but mechanisms are still poorly understood and evidence to guide clinical practice is currently inadequate.

## Introduction

Pain affects millions of people worldwide, impairs mood, social and professional life, and is often difficult to treat. There is increasing evidence that the microbiota-gut-brain axis has a pivotal role in the development and modulation of the central nervous system (CNS) and gastrointestinal functions (1).

The microbiota-gut-brain interaction can modulate stress and pain perception and afferent sensory pathways, thus playing a crucial role in the control of behaviors and different neuropsychiatric disorders (2).

Alteration of gut microbiota (dysbiosis) has been demonstrated in many conditions in which pain is a key manifestation. Thus, the likely correlation between changes in gut microbiota and functional gastrointestinal disorders (FGIDs) could provide preventative as well as therapeutic options in adults and children (3). In fact, dietary interventions and probiotics can modify the composition and function of the gut microbiota, potentially providing a useful approach in several gastrointestinal conditions (4).

Many studies showed that probiotics could have both nutritional and immunomodulatory benefits (5), and that they are potentially useful for preventing and treating numerous intestinal disorders correlated to changes in gut microbiota resulting from a variety of factors (e.g., diet, antibiotics, lifestyle) (6).

In addition, specific strains of probiotics have been shown to be able to affect the intestinal microbiota, have anti-inflammatory properties (7) and modulate visceral hypersensitivity (8), thus improving abdominal pain management.

## Methods

This narrative review was conducted searching scientific databases for articles reporting on probiotics, perception of pain, and FGIDs in pediatric age.

The search was performed in PubMed, Medline, Embase, Cochrane library, and Web of Science.

The following subject MeSH headings were used: “Probiotics” [Mesh], “Newborns, infants, children [MeSH], “Functional abdominal pain [MeSH], “Functional gastrointestinal disorders” [MeSH], “Infantile colic” [Mesh], “Irritable bowel syndrome” [MeSH], “Constipation” [MeSH], “Gastroesophageal reflux” [MeSH]. Proper Boolean operators such as “AND” and “OR” were also included.

Additional studies were added using references of articles taken from the mentioned databases. Search limits were set for randomized placebo-controlled clinical trials (RCT), written in English, conducted only on human subjects, and published between January 2011 and September 2021.

### Gut-Brain Axis and Nociception

The gut-brain interaction is a very complex bidirectional communication between the CNS and the gastrointestinal system (9) and represents a key modulator of human health (10).

It correlates in a bidirectional communication cognitive and emotional centers in the CNS, neuroendocrine and neuroimmune systems, sympathetic and parasympathetic systems, the hypothalamic-pituitary-adrenal axis, and the gut microbiota. On the other hand, gut microbiota may also modulate the gut-brain interactions, creating the so called microbiota-gut-brain axis (11).

Gut microbiota is the set of synbiotic microorganisms that coexist with the human organism providing genetic and metabolic substrates, fundamental to human nutrition and homeostasis (12, 13). Nonetheless, an imbalance of this complex relationship between microbiota, gut and brain can alter both the central and peripheral pathways associated with the perception and manifestation of pain (14).

While the pathogenesis and perception of somatic pain are fairly well-understood, visceral pain and its pathogenetic mechanisms are not fully known; therefore, an adequate therapeutic intervention represents a complex challenge.

The gut microbiota may modulate visceral pain perception and nociception and presents an important correlation with visceral function and autonomic and emotional reactions. Thus, gut microbiota could represent a possible target for new therapeutic strategies against visceral and abdominal pain (1–3). Some factors, such as diet, prebiotics, and probiotics, could modulate the gut microbiota, thus presenting a possible role in pain management and overall wellbeing (6–8).

### Probiotics and Gut Microbiota

Probiotics are defined by the World Health Organization (WHO) (15) as “live microorganisms which when administered in adequate amounts confer a health benefit on the host.” Noteworthy, to be defined as such they should demonstrate evidence-based health effects (16).

Probiotics appear to be useful in preventing and/or treating many gastrointestinal disorders, such as infectious and antibiotic-associated diarrhea, ulcerative colitis, infantile colic, irritable bowel syndrome (IBS), and functional abdominal pain (10, 17, 18). They interact with the human host in different ways and at multiple levels: mucus and epithelial layers, lamina propria, gut-associated lymphoid tissue (GALT).

The activity of probiotics is strain and species-specific and can change according to the physiology and eating habits of different subjects (19). Specific probiotics can directly act on gut motility and barrier functions, host digestion, immune responses, nociception, metabolism, behavior, and microbiota composition (16, 17).

Therefore, recently there has been a growing interest in the possibility of modulating the gut microbiome to improve the health of the gastrointestinal system (20, 21).

The gut microbiota plays a central role in maintaining the guest's wellbeing. Understanding its impact on individual health is fundamental to elaborate targeted strategies for its modulation, especially when dysbiosis is present as is often the case in various chronic gastrointestinal disorders (16). Hence, modulating the gut microbiota composition and function with probiotics that have a proven efficacy for the specific condition, appears to be a logical option, both for prevention and for treatment.

### Pediatric Functional Gastrointestinal Disorders

Functional gastrointestinal disorders (FGIDs) represent a variable set of chronic or recurrent gastrointestinal symptoms without an underlying organic disease. According to the Rome IV Criteria, they represent brain-gut interaction disorders, characterized by various gastrointestinal symptoms related to motility disorders, visceral hypersensitivity, alterations of immune and mucosal function, alterations of gut microbiota and/or CNS processing disorders (22).

Functional gastrointestinal disorders occur in nearly half of healthy infants, with colic and regurgitation having a high prevalence in the first months of life and in selected populations (23, 24). In subsequent ages, FGIDs often compromise the quality of life of the affected children and their parents, with potential short and long-term consequences on the wellbeing of the whole family (25).

#### Infantile Colic

According to Rome IV Criteria, infantile colic is a FGID defined as “paroxysms of irritability, fussing or crying that starts and stops without an apparent cause, in infants younger than 4 months of age and without failure to thrive.” These episodes have to last 3 or more hours per day and occur at least 3 days per week for at least 1 week (26).

Infantile colic represents a self-limited condition, but continues to remain a major cause of concern for parents and of distress for infants (27). Recently, a large Italian prospective study recruiting infants since birth and monitoring up to 1 year of life, showed a high incidence of colic (50.7%) particularly expressed in infants born preterm, with low birth weight or exposed to antibiotics in the perinatal period (28, 29).

Of note, infants suffering from infantile colic are more likely to develop abdominal pain-related FGIDs later in life (30, 31). Moreover, infantile colic has been related to numerous medical visits and interventions (32), parental deprivation of sleep, depression, anxiety and exhaustion, and also reduced work efficiency (33, 34).

Several factors contribute to the manifestation of colic, such as genetic factors, early stressful events or trauma, alterations in intestinal motility, visceral hyperalgesia, intestinal inflammation, gut microbiota, psychosocial factors, altered parental coping.

In the last decades, different approaches to prevent and treat infantile colic have been attempted without conclusive results (35). Probiotics have been widely proposed in managing infantile colic (32, 36, 37), although their exact mechanism of action in this disorder remains poorly understood.

To date there are only few recommendations for reducing episodes of excessive crying in colicky neonate (38). Several drugs have been tried to prevent infantile colic, like antispasmodic molecules (e.g., dicyclomine) but since they may present serious adverse effects up to coma, their use in infants is not allowed.

Infants with colic have interesting differences in gut microbiota compared to infants without colic (39). A recent systematic review analyzed probiotics for the management and prevention of infantile colic. Healthy full-term infants without congenital malformations or severe diseases, with normal birth weight and normal growth rate, and without recent antibiotic or probiotic treatment, were evaluated. In this review, 6 RCTs evaluated the efficacy of *L. reuteri* DSM 17938 in breastfed infants, showing a significant reduction in crying and fussing compared to placebo (40, 41).

A randomized, double-blinded, placebo-controlled trial was conducted by Savino et al. (39) to verify the effectiveness on infantile colic of oral administration of *Bifidobacterium longum* CECT7894 (KABP042) and Pediococcus pentosaceus CECT8330 (KABP041) mix (1 × 10^9^ colony forming units). The crying/fussing time and the frequency of the crying/fussing episodes were significantly lower in the probiotics group compared to the placebo group on days 7, 14 and 21. Furthermore, infants who had taken oral probiotics presented lower fecal frequency/day compared to subjects who had taken placebo.

In 2018, Baldassarre et al. conducted a RCT in breastfed term infants using a specific multi-strain probiotic preparation (Vivomixx): a medium chain triglycerides oil suspension with four different strains of lactobacilli (*L. Paracasei* DSM 24733, *L. plantarum* DSM 24730, *L. acidophilus* DSM 24735, and *L. delbrueckii* subsp. bulgaricus DSM 24734), three strains of bifidobacteria (*B. longum* DSM 24736, *B. breve* DSM 24732, and *B. infantis* DSM 24737), and one strain of *Streptococcus thermophilus* DSM 24731 (42). Expected dose was ten drops of the study product, corresponding to 5 billion colony-forming units (CFU) of this multi-strain preparation (42). The total average crying minutes during the duration of the study (21 days) were much lower and the family quality of life on day 14 and day 21 was better in the probiotic group than in the placebo group, with a statistically significant difference. No difference emerged between the probiotic group and the placebo group in relation to stool consistency, bowel movements, and growth. Both probiotics and placebo were well-tolerated and there were no adverse events.

Previously, Roos et al. conducted a RCT in which they evaluated the stools of colicky infants after administration of *L. reuteri* DSM17938 or placebo, finding a significant correlation between reduction of symptoms and increase of Bacteroidetes (43). In this regard, a recent meta-analysis showed that colicky infants supplemented with *L. reuteri* DSM179389 presented shorter crying and/or fussing duration (40).

However, the role of probiotics in formula-fed infants with colic needs more research. Data from main infantile colic studies are summarized in Table 1.

**Table 1:** Infantile colic.

**References**	**Type of study**	**Sample size (*n*)**	**Intervention**	**Outcomes**
Sung et al. (40)	Meta-analysis	345 4–8 weeks (median age)	*L. reuteri* DSM17938 vs. placebo	Less crying and/or fussing time in breastfed infants Intervention effects insignificant in formula-fed infants
Simonson et al. (41)	Systematic review		*L. reuteri* DSM 17938 vs. placebo	50% reduction in crying time compared with placebo in breastfed infants Efficacy in formula-fed infants needs further study
Baldassarre et al. (42)	Double-blind, randomized, placebo-controlled trial	53 30–90 days	Vivomixx ^*^ vs. placebo in breastfed infants	Reduction of crying times of ≥50% from baseline on day 14 and 21 in exclusively breastfed infants
Roos et al. (43)	Randomized DBPC Trial	29 10–60 days	*L. reuteri* DSM 17938 vs. placebo	Significant correlation between reduction of daily crying time and increase of Bacteroidetes in fecal samples

* *Vivomixx (Visbiome, DeSimone Formulation): L. paracasei DSM 24733, L. plantarum DSM 24730, L. acidophilus DSM 24735, and L. delbrueckii subsp. bulgaricus DSM 24734, B. longum DSM 24736, B. breve DSM 24732, and B. infantis DSM 24737, Streptococcus thermophilus DSM 24731*.

#### Irritable Bowel Syndrome

Irritable bowel syndrome (IBS) is a FGID characterized by the association of abdominal pain with alterations in bowel habits (either diarrhea or constipation) and whose etiopathogenesis remains unclear (44–46). Several factors have been implicated, such as visceral hypersensitivity (47), gastrointestinal microbiota alterations (48), and chronic immune activation, resulting in a mild mucosal inflammation (49).

According to the biopsychosocial model, a combination of factors (e.g., genetic predisposition, early adverse events or trauma, psychological factors, gastrointestinal infections) induce changes in the enteric nervous system, resulting in alterations in gastrointestinal motor, sensory, mucosal barrier, and secretory responses (44).

To date there are no specific therapies for IBS but probiotics have long been proposed to modify the gastrointestinal microbiota (50), to modulate visceral hypersensitivity (51) and to reduce the inflammatory state (52), therefore improving symptoms and pain management. Only a limited number of RCTs testing a few probiotic strains in children with IBS have been published.

In a double-blinded, cross-over, placebo-controlled RCT, Guandalini et al. evaluated the action of the probiotic mixture VSL#3 (a formulation currently available as Vivomixx in Europe and Visbiome in the US) in 59 infants with IBS. This preparation provides 450 billion of CFU bacteria per sachet, with 8 different strains (*Bifidobacterium breve, Bifidobacterium longum, Bifidobacterium infantis, Lactobacillus acidophilus, Lactobacillus plantarum, Lactobacillus casei, Lactobacillus bulgaris*, and *Streptococcus thermophilus*). In this study, patients with on probiotics presented a significantly better score for abdominal pain/discomfort and for bloating/gassiness, with a consequent general satisfaction of caregivers (53).

In a 2014 systematic review and meta-analysis (54) *Lactobacillus rhamnosus* GG ATCC53103 (LGG), *L. reuteri* DSM 17 938 and VSL#3 were found to be more effective than placebo in relieving functional abdominal pain and IBS in pediatric age (54).

It is also plausible that an effect of probiotics on reducing intestinal permeability (shown for both LGG and VSL#3) (55) plays a role, in addition to a possible effect on gut–brain axis (56).

Of interest, administration of *L. reuteri* DSM 17938 might have a lasting effect, as its benefit on abdominal pain intensity persisted even after its discontinuation (57).

A 2017 study showed in addition that *L. reuteri* DSM 17938 was better than placebo in improving the normal activities of children with IBS and their parents (58). A systematic review and meta-analysis in 2020 concluded that this probiotics was able to reduce perception of pain in children with functional abdominal pain (59).

Also LGG showed better efficacy than placebo both in children with functional abdominal pain alone and in those with IBS (60).

While specific strains of probiotics appear, as we have seen, to reduce IBS-related pain (61, 62), in terms of prevention of gastrointestinal disorders in children, a 2019 review concluded that there is insufficient evidence to recommend their use for the prevention of any functional gastrointestinal disorder (63).

To summarize data on probiotics in IBS in children, some specific strains or multi-strain preparations of probiotics have shown efficacy and can be therefore considered a potential therapeutic option, also in consideration of their excellent safety profile (64) and the very limited therapeutic armamentarium available. However, due to heterogeneity of study design and the scarcity of randomized clinical trials available in pediatric age, there is an obvious need for more large, placebo-controlled trials in order to reach solid evidence to recommend probiotic administration for IBS in pediatric age. Table 2 summarized data from main studies on IBS in pediatric age.

**Table 2:** Irritable bowel syndrome.

**Reference**	**Type of study**	**Sample size (*n*)**	**Intervention**	**Outcomes**
Guandalini et al. (54)	Double-blinded, placebo-controlled RCT	59 4–18 years	VSL#3^*^ vs. placebo for 6 weeks, with controls every 2 weeks.	VSL#3 significantly superior in the subjective assessment of relief of symptoms, with better score for abdominal pain/discomfort, bloating/gassiness, and general satisfaction of caregivers
Romano et al. (58)	Double-blinded, placebo-controlled RCT	60 6–16 years	*L. reuteri* DSM 17938 vs. placebo	*L. reuteri* DSM 17938 related to significantly lower pain intensity compared with the placebo controls. Lasting effect over time: persistent decrease in abdominal pain intensity even after discontinuation of the probiotic
Maragkoudaki et al. (59)	Double-blinded, placebo-controlled RCT	54 5–16 years	*L. reuteri* vs. placebo	Both *L. reuteri* and the placebo effective in alleviating pain, but only *L. reuteri*, improved the child's and family's normal activities
Trivić et al. (60)	Systematic review and meta-analysis	641 4–18 years	*Lactobacillus rhamnosus* GG and *Lactobacillus reuteri* DSM 17938 vs. placebo	*L. reuteri* DSM 17938 related to significant reduction in pain intensity and increase in number of days without pain
Horvath et al. (61)	Meta-analysis	290 5–17 years	*L. rhamnosus* GG ATCC53103 vs. placebo	*L. rhamnosus* GG moderately improve abdominal pain-related FGID, particularly among children with IBS

* *VSL#3: Vivomixx (Visbiome, DeSimone Formulation): 8 different strains (Bifidobacterium breve, Bifidobacterium longum, Bifidobacterium infantis, Lactobacillus acidophilus, Lactobacillus plantarum, Lactobacillus casei, Lactobacillus bulgaris, and Streptococcus thermophilus)*.

#### Constipation

According to Rome IV criteria (26, 65), constipation is one of the most common functional gastrointestinal disorders in pediatric population (66) and is often associated with abdominal pain.

The principal pathogenic mechanism of constipation is a dysregulated or deficient colonic propulsive motor pattern (67) and the prolonged fecal stasis may impact on gut microbiota further impairing motility (68).

Several therapeutic options do exist for constipation: fiber supplements, osmotic agents, laxatives; but their effect is not always optimal, and their prolonged administration is faced with difficulties by both the children and their parents. Hence, probiotics have been tried as a potentially useful and safe alternative for this condition. In fact, probiotics are believed to improve peristalsis and reduce intestinal stasis (69) by modifying the gut microbiota, increasing the production of lactate and short-chain fatty acids and reducing luminal pH.

Although some strains (e.g., *L. casei* rhamnosus Lcr35) have been shown to reduce the passage of hard stools, no evidence of efficacy regarding frequency of evacuation, fecal incontinency, and abdominal pain have been demonstrated.

Different systematic reviews and meta-analysis concluded that there is not enough evidence for the systematic recommendation of probiotics for this indication (70–72). Also the European (ESPGHAN) and the North American (NASPGHAN) Societies of Pediatric Gastroenterology, Hepatology and Nutrition do not recommend probiotics in the management of functional constipation in pediatrics (73). Table 3 summarizes data relating to constipation.

**Table 3:** Constipation.

**First author**	**Type of study**	**Sample size (*n*)**	**Intervention**	**Outcomes**
Huang et al. (70)	Systematic review and meta-analysis	498 <18 years	Different probiotic strains tested in different studies (*L. rhamnosus, L. casei, S. thermophilus, B. breve, L. acidophilus, B. infantis, L. sporogenes*)	Probiotics significantly increased the stool frequency
Wojtyniak et al. (72)	Systematic review	515 6 months to 16 years	*L. rhamnosus* casei Lcr35 vs. placebo Other probiotics studied in single trials (*L. rhamnosus* GG, *L. reuteri* DSM 17938, *B. lactis* DN-173 010, *S. thermophilus* CNCM I-1630, *B. longum*, Protexin^*^)	No difference regarding frequency of fecal incontinence or abdominal pain. No evidence to recommend probiotics in constipation.
San Gomes et al. (73)	Systematic review	564 < 19 years	Different probiotic strains evaluated (*L. rhamnosus* GG, L. *casei* rhamnosus Lcr35, *L. reuteri, B. lactis, B. longum*, Protexin^*^, Probiotic mix^**^)	No evidence to recommend probiotics in the treatment of constipation in pediatrics

* *Protexin: L. casei PXN 37, L. rhamnosus PXN 54, S. thermophiles PXN 66, Brief bifidobacterium PXN 25, L. acidophilus PXN 35, B. infantis PXN 27 and L. bulgaricus PXN 39*.

** *Probiotic mix: Brief bifidobacterium M-16 V, Infant Bifidobacterium M-63 and Bifidobacterium longum BB536*.

Similar to other conditions, it would be useful to standardize criteria, definitions, and outcomes to evaluate the therapeutic action of probiotics in large and homogeneous pediatric populations. (74, 75).

#### Gastroesophageal Reflux

Gastroesophageal reflux disease (GERD) represents a complex of symptoms that compromise the quality of life or complications caused by the retrograde flow of gastric contents into the esophagus and/or respiratory tract, as defined by the World Gastroenterology Organization (76).

Among the wide spectrum of manifestation, GERD may cause heartburn and epigastric or retro-sternal pain.

The prevalence varies between 8 and 33%, depending on age group, countries, selection of patients, and diagnostic criteria (77).

Currently, proton-pump inhibitors (PPIs) are the first-choice treatment for GERD (78), but long-term use of PPI can modify gut bacterial population and suppress the gastric acid barrier, determining dysbiosis that may contribute to abdominal pain (79, 80).

Specific strains of probiotics may reduce the adverse effects of PPI on gut microbiota although their effects in subjects with dyspepsia and GERD symptoms have not been properly investigated (81) and current evidence of efficacy is insufficient to provide any recommendation (82).

In 2017 Vandenplas et al. showed that a synbiotic infant formula supplemented with *B. lactis* and fructo-oligosaccharides resulted in a lower incidence of daily regurgitations (83).

Specific probiotic strains, in particular *L. reuteri* DSM17938, could improve functional symptoms of esophagus and stomach promoting gastric emptying and reducing the number of episodes of regurgitations per day (63). Table 4 summarizes data relating to gastroesophageal reflux and GERD.

**Table 4:** Gastroesophageal reflux.

**Reference**	**Type of study**	**Sample size (*n*)**	**Intervention**	**Outcomes**
Depoorter et al. (72)	Review	951	Different probiotic strains evaluated (*L. reuteri* DSM 17938, *Bifidobacterium lactis*)	Reduction daily regurgitation
Cheng et al. (82)	Systematic review	918	Different probiotic strains evaluated (*B. bifidum* W23, *B. lactis* W52, *B. longum* W108, *L. casei* W79, *L. plantarum* W62, *L. rhamnosus* W71, *L. reuteri, L. rhamnosus* GG, *S. boulardii, L. gasseri* LG21, *B. bifidum* YIT 1034, *B. lactis* HN019, *L. acidophilus* La5, *B. lactis* Bb-12, *Lactobacillus bulgaricus, Lactobacilus paracasei, Streptococcus thermophilus*)	Insufficient evidence to recommend regular administration of some specific probiotics for GERD
Vandenplas et al. (83)	Prospective open trial	280	*B. lactis* and fructo-oligosaccharides	Lower incidence of daily regurgitation

More studies with a greater number of infants and well-defined endpoints may clarify the possible role of probiotics in GERD, currently unclear at best.

## Conclusions

Painful conditions are strongly disabling at all ages but are often difficult to treat. Pain is one of the most common symptoms in children with gut barrier dysfunction, dysbiosis, mucosal inflammation, and dysmotility.

Gut microbiota seems to have a central role in multiple aspects of human health and diseases. Different factors including genes, stress, diet, antibiotic therapy, infections, early life events and lifestyle may alter the composition of the microbiota; therefore, it is conceivable that well-selected probiotics might reverse this detrimental effect.

Many studies have reported reduction of abdominal pain in children with infantile colic and IBS when specific strains of probiotics, as pointed out in the narrative, are administered. However, several limitations (e.g., heterogeneity of the studies, small sample size, different strains, various treatment options) impair the assessment of efficacy of probiotics on abdominal pain in children.

Further clinical studies should preferably analyze both principal clinical outcomes and composition and function of gut microbiota.

The development of a minimum core outcome set for clinical research in children with functional gastrointestinal disorders would be desirable to compare the different therapeutic interventions and the results between studies. Properly designed, randomized, double-blind, placebo-controlled studies with a sufficient number of participants, well-defined endpoints and a longer duration are needed.

## Author Contributions

MC and MB conceptualized and designed the study, drafted the initial manuscript, and revised the manuscript. VR and MC led the data acquisition and interpretation and revised the manuscript. NL, MB, SG, and SS made substantial contributions to the conception of the study and reviewed the manuscript. All authors conceived and designed the study protocol. All authors have read and agreed to the published version of the manuscript.

## Conflict of Interest

The authors declare that the research was conducted in the absence of any commercial or financial relationships that could be construed as a potential conflict of interest.

## Publisher's Note

All claims expressed in this article are solely those of the authors and do not necessarily represent those of their affiliated organizations, or those of the publisher, the editors and the reviewers. Any product that may be evaluated in this article, or claim that may be made by its manufacturer, is not guaranteed or endorsed by the publisher.

## Abbreviations

CNS: Central Nervous System
FGIDs: Functional Gastrointestinal Disorders
ADD: Antibiotic-Associated Diarrhea
GI: Gastrointestinal
RCT: randomized clinical trials
WHO: World Health Organization
IG: intervention group
PG: placebo group
IBS: Irritable Bowel Syndrome
GALT: Gut-Associated Lymphoid Tissue
GERD: Gastroesophageal Reflux Disease
PPIs: Proton-Pump Inhibitors
LGG: *Lactobacillus rhamnosus* GG
TNF-α: Tumor Necrosis Factor-α.
